The article "Differential Diagnosis of Preinvasive Lesions in Small Pulmonary Nodules by Dual Source Computed Tomography Imaging" was published in 2022. Journal: Comput Math Methods Med.

# Differential Diagnosis of Preinvasive Lesions in Small Pulmonary Nodules by Dual Source Computed Tomography Imaging

**DOI:** 10.1155/2022/6255024

**Published:** 2022-07-04

**Authors:** Hongjun Yan, Ye Hua, Tingcui Zhang, Wen Liu

**Affiliations:** ^1^Image Center, The First People Hospital of Baiyin, Baiyin, 730900 Gansu, China; ^2^Operation Room, Gaotang People's Hospital, Gaotang, Shandong, China; ^3^Department of Party-Masses Work, The First People Hospital of Baiyin, Baiyin, 730900 Gansu, China; ^4^Department of Imaging, Yulin First Hospital, Yulin, 718000 Shaanxi, China

## Abstract

This study was aimed to explore the differential diagnosis value of preinvasive lesions/minimally invasive adenocarcinoma and invasive adenocarcinoma manifesting as small pulmonary nodules under dual source computed tomography (DSCT) imaging. The patients with nodular manifestations of adenocarcinoma in situ (AIS)/microinfiltrating adenocarcinoma (MIA) were selected as group X, including 14 cases. A total of 31 cases with nodular infiltrating adenocarcinoma were selected as group Y. The enhanced dual-energy image obtained by DSCT dual-energy scan was transferred to the software to obtain the energy image and iodine distribution map. SPSS 18.0 was used for statistical analysis. *P* < 0.05 was considered statistically significant. All measurements were labeled as mean *x͞*±*S* standard deviation. In the CT findings of microinfiltrating adenocarcinoma and infiltrating adenocarcinoma, lobulation sign, burr sign, vacuole sign, and pleural depression sign can help the diagnosis of infiltrating adenocarcinoma. The results showed that lobulation sign, burr sign, vacuole sign, and pleural depression sign could be used as the distinguishing feature of preinvasive lesion/microinvasive adenocarcinoma and invasive adenocarcinoma. Receiver-operating characteristic (ROC) curve analysis showed that the critical value, sensitivity, and specificity of lesion diameter ≥1.4 cm and CT value ≥14.14HU for diagnosis of invasive lung adenocarcinoma were 1.32 and 14.14, 88.4% and 94.4%, and 67.3% and 75.8%, respectively. There were substantial differences in CT values between the two groups under low energy level (42-99 kev) (*P* < 0.05). DSCT dual-energy imaging can quantitatively identify preinvasive pulmonary nodules with multiple parameters.

## 1. Introduction

Lung cancer is one of the most common malignant tumors in the lung. In recent years, the incidence and mortality of lung cancer have been very high, and people pay great attention to it. The incidence of lung cancer varies greatly in different countries and regions. In recent years, the incidence of lung cancer in China is also rising and has become the highest incidence of cancer in men and the second highest incidence of cancer in women. Lung adenocarcinoma is the most common type of lung cancer, accounting for 43.7%-47.1% [1]. The incidence of lung adenocarcinoma is increasing gradually. There are many factors to determine the malignant degree of lung adenocarcinoma, among which the pathological grade of adenocarcinoma is an independent index to judge the malignant degree of lung adenocarcinoma. Studies pointed out that compared with moderately and highly differentiated lung adenocarcinoma, poorly differentiated lung adenocarcinoma has a lower postoperative survival rate and a higher postoperative local recurrence rate, and is more likely to occur lymph node metastasis and distant metastasis [2]. Therefore, different grades of lung adenocarcinoma have different histological features and prognosis. Preoperative noninvasive understanding of the pathological grade of lung adenocarcinoma has great influence on the prognosis of lung cancer and the selection of treatment. Dual source computer tomography (DSCT) dual-energy imaging is a novel imaging technology, featuring fast imaging speed and low radiation dose [3]. Its imaging model provides a new multiparameter diagnostic model for lesion analysis, achieving the separation and identification of substances. The iodine map can measure the iodine content in any region and better reflect the perfusion of tissues than conventional CT enhancement [4]. DSCT dual-energy imaging can express chemical information of substances by tracing energy spectrum curve, identify different chemical substances (such as ligaments and topout), and obtain the effective atomic number, iodine group diagram, and aquarium diagram of any tissue, providing a new idea for benign and malignant differentiation of tumors [5].

The article "Differential Diagnosis of Preinvasive Lesions in Small Pulmonary Nodules by Dual Source Computed Tomography Imaging" was published in 2022. Journal: Comput Math Methods Med.

Currently, imaging explorations on lung adenocarcinoma mainly focus on nodule morphology, energy spectrum blood supply, and lesion differentiation degree. In the CT differential diagnosis of preinvasive lesions (PL) and invasive lung adenocarcinoma, studies found that there is statistically substantial difference between preinvasive lesions and solid parts of invasive lung adenocarcinoma (*P* < 0.005) [6]. The maximum diameter of the lesion increased from anterior to invasive adenocarcinoma (*P* < 0.005). Studies also suggested that the optimal diameter limit for high-resolution CT to distinguish AAH/AIS and IAC is 110 mm, with sensitivity of 95.6% and specificity of 46.7% [7]. Therefore, it is believed that the lesion size and CT value can reflect the invasion of the lesion, that is, the larger the lesion, the higher the CT value and the deeper the invasion. Energy spectrum CT material analysis technology can quantitatively analyze the changes of lung tumor blood supply and can make differential diagnosis of different types of tumors. The degree of enhancement is related to microvascular density. The more blood vessels the tumor supplies, the greater the degree of enhancement and the higher the iodine content [8]. Iodine content can reflect the blood supply status of lesions. Currently, there are few literature reports on differential diagnosis of microinvasive adenocarcinoma and invasive adenocarcinoma with pulmonary nodules in preinvasive lesions by energy spectrum CT [9, 10]. The blood supply and differentiation degree of lung adenocarcinoma on energy spectrum CT also provide theoretical basis for this study. In this study, DSCT imaging was used to investigate the differential diagnosis value of preinfiltrating lesions (microinfiltrating adenocarcinoma) and infiltrating adenocarcinoma (infiltrating adenocarcinoma). Multiparameter and quantitative identification of pulmonary nodular preinfiltration lesions was expected to bring significance to clinical application.

## 2. Materials and Methods

### 2.1. Research Objects

The patients who received conventional 62-row DSCT from January 2018 to November 2020 in the hospital were included as the study subjects. Inclusion criteria: (i) patients with lung adenocarcinoma with single nodule diameter ≤2.9 cm; (ii) the density of pulmonary nodules was relatively uniform, without substantial calcification, necrosis, or cavity, and the solid range was sufficient for measurement; (iii) no radiotherapy, chemotherapy, or interventional therapy; (iv) the image data was complete. Exclusion criteria: (i) allergic history of iodine contrast agent, severe heart, liver, and renal insufficiency; (ii) thyroid dysfunction; (iii) a history of other concomitant tumors; (iv) cystic ground glass appearance of lung cancer lesions. A total of 45 patients were eligible for lung adenocarcinoma. Based on pathological findings and international multidisciplinary typing in 2011, patients with nodular manifestations of adenocarcinoma in situ (AIS)/microinfiltrating adenocarcinoma (MIA) were selected as group X, including 14 cases. A total of 31 cases with nodular infiltrating adenocarcinoma were selected as group Y. This study had been approved by the ethics committee of the hospital, and all the families of patients included in the study signed informed consent.

### 2.2. Equipment and Methods

62-layer dual source scanner was used. As for the enhanced CT scan, the dual source Liver VNC sequence was adopted, and the A-Ball and B-Ball tubes acquired images at the same time. Scanning parameters were matrix =514 × 514, A tube =142 kV, 82mAs; B tube =102 kV, 162mAs. The real-time dynamic exposure dose was CARE Dose 4D at the beginning, the detector width was 30 × 0.5 mm, and the spacing was 0.6 mm. The reconstruction parameters were as follows. The layer spacing was 1.2 mm, the layer thickness was 1.6 mm, and the reconstruction function was D24f. Three sets of images with 102 kV, 142 kV, and linear fusion (fusion coefficient =0.29, equivalent to 124 kV) were obtained. 82 mL of nonionic iodine contrast medium (iohexol 304 mg I/mL) was injected through the median cubital vein via a double-barrel high-pressure syringe for enhanced scanning. The flow rate was 3.1 mL/s, and the total amount was 1.2 mL/Kg body weight. After injection, 32 mL of normal saline was injected at the same flow rate. The contrast agent group injection tracking software was employed to trigger the scan start, and the arterial phase trigger threshold was 102HU. Scanning and image acquisition were started at 26 s and 29 s after contrast injection in the arterial and venous phases, respectively.

The article "Differential Diagnosis of Preinvasive Lesions in Small Pulmonary Nodules by Dual Source Computed Tomography Imaging" was published in 2022. Journal: Comput Math Methods Med.

The location, size, CT value, presence, or absence of lobulation sign, burr sign, vacuole sign, bronchiectasis sign, pleural depression sign, and vascular cluster sign were observed and measured on conventional CT plain scan. The flat scan and enhanced Mono images of 42-188 kev (10 keV interval) were extracted by the energy spectrum analysis software, and the corresponding energy decay curves in the arteriovenous phase were plotted for each. The resulting curves were analyzed and compared in the same coordinate system. The mean energy decay curves of the arterial and venous phases of lung adenocarcinoma were plotted by taking the mean absolute CT of 42-188 kev under all energy decay curves. Arterial and venous iodine content of all tumor lesions was measured. To reduce the influence of patient weight and vascular factors on this study, all measured primary iodine concentrations should be normalized to the same level of aortic iodine concentration. The normalized iodine concentration (NIC) was calculated as follows: normalized iodine concentration = initial iodine concentration/aortic iodine concentration in the same layer.

### 2.3. Image Postprocessing

Image analysis and measurement were performed using DSCT-specific dual-energy software. After the dynamic phase and venous phase energy images were transferred to the dual-energy software, they were, respectively, transferred to the dual-energy card of Multi-Modality workstation and adjusted to the default parameter values. The “Liver VNC” model was adopted to adjust the fusion rate of CT and iodinated contrast agent under the mediastinal window. The fusion rate of the iodine contrast agent was adjusted to 100%, and the distribution images of iodine in the arteriovenous and arterial phases were obtained (Figure 1). The arterial and venous phases were in single-energy mode. By moving the single-energy (KEV) axis, a series of single-energy images of 42-188 keV were obtained. Every nine energy cells were selected one by one, and a single-energy image was saved. Next, a region of interest (ROI) was selected from a single-energy image under each Kev, the CT value of the lung nodule was measured, and an energy spectrum curve was then plotted.

The article "Differential Diagnosis of Preinvasive Lesions in Small Pulmonary Nodules by Dual Source Computed Tomography Imaging" was published in 2022. Journal: Comput Math Methods Med.

### 2.4. Observation Indicators

The location, size, CT scan value, presence, or absence of lobulation sign, burr sign, vacuole sign, bronchial air sign, pleural depression sign, vascular cluster sign, single-energy CT value, and iodine concentration of each case were collected. The nodules were round or irregular dense opacities with a maximum diameter of ≤2.9 cm. The lobulation sign refers to the uneven margins of the lesion due to the inconsistent growth rate of the tumor in all directions. In the burr sign, tumor cells and tumor stroma infiltrate in all directions, stimulate the proliferation of surrounding connective tissue, and form straight, long, or short burrs. Air bronchi sign refers to the bright bronchial shadows visible in the lesions of lung tissue. The vacuolar sign refers to the appearance of a small focal light-transmitting area with a diameter less than 4.8 mm in the nodule. Pleural depression syndrome refers to a lung lesion adjacent to the visceral pleura that exhibits an angular depression in cross-section with the tip pointing toward the lesion. Vascular plexus syndrome is a reactive fibrous connective tissue hyperplasia that pulls adjacent vessels toward or into the nodule.

### 2.5. Statistical Analysis

SPSS 22.0 was used for statistical analysis of all data, and *P* < 0.05 was considered statistically significant. Four table chi-square test was used to compare the CT findings of preinvasive lesions with microinvasive adenocarcinoma and invasive adenocarcinoma. Two-independent sample *T* tests were used to compare the size and CT density of invasive adenocarcinoma and preinvasive/microinvasive adenocarcinoma. Normalized iodine concentration (NIC) and CT spectral characteristics of invasive adenocarcinoma and preinvasive/microinvasive adenocarcinoma were compared by *T* test of two independent samples. The two-independent sample *T*-test inferred whether the mean values of two independent populations from two samples were significantly different based on the sample data. All measurements were labeled as mean plus or minus standard deviation. The receiver-operating characteristic (ROC) curve was plotted to determine the diagnostic thresholds, CT values, and standardized iodine content of preinvasive lesions, microinvasive adenocarcinoma, and invasive adenocarcinoma.

The article "Differential Diagnosis of Preinvasive Lesions in Small Pulmonary Nodules by Dual Source Computed Tomography Imaging" was published in 2022. Journal: Comput Math Methods Med.

## 3. Results

### 3.1. Clinical Features

A total of 45 patients were included in this study, including 20 females and 25 males, ranging in age from 27 to 79 years old, with an average age of 57.79 years. All patients underwent surgical resection, pathologically confirmed lung adenocarcinoma, and 45 tumor nodules were obtained. In Figure 2, there were 31 cases of invasive adenocarcinoma with an average age of 57.41. There were 5 cases of preinvasive lesions (all AIS) and 9 cases of minimally invasive adenocarcinoma. The average age of preinvasive lesions/minimally invasive adenocarcinoma was 56.39. As for the clinical symptoms, there were no symptoms in 10 cases, fever in 8 cases, cough in 14 cases, chest pain in 12 cases, chest tightness in 15 cases, blood in sputum in 9 cases, and smoking history in 18 cases. According to the new classification criteria for lung adenocarcinoma proposed by the *International Association for Research Lung Cancer/European Respiratory/American Thoracic Society* (IASLC/Human/ATS) shown in Table 1, the associated clinically meaningful survival between AIS and MIA was 100% or close to 100%. 14 AIS/MIA patients with nodular manifestations were selected as group X and 31 nodular invasive adenocarcinomas in group Y.

### 3.2. Results of DSCT Imaging Examination

After DSCT scanning, the morphological comparison of the CT image features of the X and Y groups was performed.  Figure 3 shows that in the two groups of patients, the occurrence probability of lobulation sign, burr sign, vacuole sign, and pleural depression sign in group Y was higher than that in group X, and the difference between the two groups was statistically substantial (*P* < 0.05).

The nodule size and CT value were compared between the X group and the Y group. From Figure 4, the nodule sizes of patients in group X and group Y were (14.33 ± 4.51) mm and (21.40 ± 3.32) mm, respectively, and the CT values were (10.14 ± 1.93) HU and (24.69 ± 3.71) HU. After comparison, it was found that the nodule size and CT value of group Y were larger than those of group X, and the difference was statistically substantial (*P* < 0.05).

The differences between the two groups of patients in the arterial and venous phases of standard iodine concentrations were then compared.  Figure 5 shows that the standard iodine concentration values in the arterial phase of patients in group X and group Y were (0.079 ± 0.022) mg/mL and (0.124 ± 0.052) mg/mL, respectively. The standard iodine concentration values in the venous phase were (0.165 ± 0.017) mg/mL and (0.332 ± 0.057) mg/mL, respectively. After comparison, it was found that the standard iodine concentration of patients in group Y in arterial phase and venous phase was always higher than that in group X, and the difference between the two groups was statistically substantial (*P* < 0.05).  Figure 6 shows the imaging features of patients with different disease types.

The article "Differential Diagnosis of Preinvasive Lesions in Small Pulmonary Nodules by Dual Source Computed Tomography Imaging" was published in 2022. Journal: Comput Math Methods Med.

### 3.3. Analysis of the Diagnostic Value of DSCT in Preinvasive Lesions of Small Pulmonary Nodules

Then, the ROC curve was drawn to compare the value of nodule size, CT value, and standard iodine concentration in diagnosing preinfiltrating lesions of small pulmonary nodules. The results are shown in Figure 7. ROC curve analysis showed that the nodule size and CT value cutoff values for diagnosing invasive lung adenocarcinoma were 1.32 and 14.14, respectively. The diagnostic sensitivity of nodule size was 88.4%, and the specificity was 67.3%. The diagnostic sensitivity of CT values was 94.4%, and the specificity was 75.8%.

Diagnosis of NIC was as follows. The standard iodine concentration was used for analysis under the ROC curve, the area under the ROC curve in the arterial phase was 0.959, the diagnostic sensitivity was 88.0%, and the specificity was 100%. The area under the ROC curve for the venous phase was 0.980, the diagnostic sensitivity was 92.34%, and the specificity was 100%. The two-phase enhanced standard iodine concentration was used to discriminate the difference between the X group and the Y group was statistically substantial (*P* < 0.05). From the area comparison, it was concluded that the standard iodine concentration value in the venous phase had the highest accuracy in diagnosing preinvasive lesions/microinvasive and adenocarcinoma-invasive adenocarcinoma.

## 4. Discussion

The basic principle of DSCT dual-energy imaging is exploring the decay law of the interaction between matter and X-rays at two different high and low energies. The energy is derived from the different X-ray attenuation values of different objects for different energies [11]. Compared with ordinary CT, spectral CT has stronger advantages because spectral CT uses single-energy images, while conventional CT is a traditional mixed-energy image. Therefore, spectral CT images can effectively reduce metal and hardening artifacts, clearly distinguish anatomical structures, reveal pathological details, and make CT values more accurate [12]. Second, spectral CT can provide multiparameter quantitative analysis, especially the iodine-based map. The main component of CT-enhanced contrast agents is iodine. The iodine-based map can clearly observe the iodine content level of the lesion and the boundary between the lesion and the surrounding tissue [13]. In addition, CT energy spectrum imaging provides visual analysis tools such as histograms, scattergrams, energy spectrum curves, water-based maps, and iodine-based maps [14]. Some studies suggested that the standard iodine concentration at the venous stage has the highest accuracy in diagnosing preinvasive lesions/micro-infiltrates and adenocarcinoma infiltrating adenocarcinoma, which is consistent with some of our research results [15] and further broadens the application platform of CT in clinical and scientific research [16]. DSCT dual-energy imaging technology provides a new diagnostic mode.

The article "Differential Diagnosis of Preinvasive Lesions in Small Pulmonary Nodules by Dual Source Computed Tomography Imaging" was published in 2022. Journal: Comput Math Methods Med.

Preinvasive lung lesions belong to precancerous lesions. Generally, they are diagnosed as precancerous lung lesions after pulmonary nodules are found by CT and pathologically confirmed by biopsy of tissue nodules under tracheoscopy or surgical resection. Therefore, attention and vigilance should be paid to them. Dual source CT dual-energy imaging technology, as a cutting-edge imaging modality, can provide multiparameter imaging for quantitative analysis of tumor morphology and functional metabolic state [17]. The qualitative and quantitative identification of preinvasive lesions/minimally invasive adenocarcinoma and invasive adenocarcinoma was performed by combining morphological features, energy spectrum curves, and NIC. The morphological and marginal features of lung adenocarcinoma on CT suggest its inherent pathological features [18]. Lung adenocarcinomas are generally round or quasi-round, reflecting a growth pattern that suggests accumulation and expansion of the lesion [19]. Lobulation is characterized by an uneven edge of the lesion, and its pathological basis is affected by the uneven growth of the surrounding lung interstitium and fibrous tissue limiting tumor growth. Relevant studies suggested that the margins of solitary malignant pulmonary nodules are mostly lobulated, and about 83% to 91% of lobulated nodules are malignant [20]. Studies revealed that lobulation sign was more prominent in invasive lung adenocarcinoma than precancerous lesions, and the difference in lobe distribution was statistically substantial (*P* < 0.05) [2]. The results showed that the incidence of lobular sign in invasive adenocarcinoma was higher than that in preinvasive adenocarcinoma and minimally invasive adenocarcinoma, and the difference between the two groups was statistically substantial (*P* < 0.05), which was consistent with the results of some studies. In this study, the CT spectra and NIC were able to judge to a certain extent to distinguish between preinvasive lesions/minimally invasive adenocarcinoma and invasive adenocarcinoma, so that the clinicians can obtain a preliminary assessment before surgery, to formulate a reasonable treatment plan for the patient and to assess the prognosis of the patient, which brings a lot of benefits. Because of the limited study time, the small number of cases collected in this study, especially in the preinvasive lesion/minimally invasive adenocarcinoma group, a detailed subtype classification of lung invasive carcinomas was not performed, so further improvements will be warranted by expanding the sample size in the future.

The article "Differential Diagnosis of Preinvasive Lesions in Small Pulmonary Nodules by Dual Source Computed Tomography Imaging" was published in 2022. Journal: Comput Math Methods Med.

## 5. Conclusion

Imaging changes such as preinvasive lesions, microinvasive adenocarcinoma, and CT findings of invasive adenocarcinoma, lobulation sign, burr sign, vacuole sign, and pleural depression are helpful for the diagnosis of invasive adenocarcinoma. The standard iodine concentration of venous phase was the most accurate for the diagnosis of preinvasion/microinvasion and adenocarcinoma infiltrating adenocarcinoma. However, there are still many problems and deficiencies in the research. In this study, the sample size was too small. More subjects should be included, not just in a single area or a small area. In conclusion, this study is of great significance for realizing early diagnosis of invasive adenocarcinoma and improving clinical treatment effect and prognosis of patients.

## Figures and Tables

**Figure 1:** Legend of iodine concentration measurement (a) in arterial phase and iodine concentration measurement (b) in venous phase.

**Figure 2:** Number of included lesions for invasive adenocarcinoma, preinvasive lesions, and minimally invasive adenocarcinoma.

**Figure 3:** Comparison of CT features of the two groups of patients. I: lobulation sign; II: burr sign; III: vacuole sign; IV: pleural depression sign. ∗Compared with X group, *P* < 0.05.

**Figure 4:** Comparison of nodule size and CT density (unenhanced scan) between the two groups of patients. ∗ Compared with X group, *P* < 0.05.

**Figure 5:** Comparison of standard iodine concentrations in the arterial and venous phases of the two groups. ∗Compared with X group, *P* < 0.05.

**Figure 6:** CT images of different types of patients. (a) Man, 57 years old, with an in-situ adenocarcinoma of the upper lobe of the right lung; (b) Man, 57 years old, with a microinvasive adenocarcinoma of the middle lobe of the right lung.

**Figure 7:** ROC curve analysis of the diagnostic efficiency of each indicator.

**Table 1:** Clinical symptoms of the included patients.

Clinical symptoms	Cases
None	10
Fever	8
Cough	14
Chest pain	12
Chest tightness	15
Blood in sputum	9
Smoking history	18

The article "Differential Diagnosis of Preinvasive Lesions in Small Pulmonary Nodules by Dual Source Computed Tomography Imaging" was published in 2022. Journal: Comput Math Methods Med.

## Data Availability

The data used to support the findings of this study are available from the corresponding author upon request.
